# Study on OBE Teaching Concept in the Context of Deep Learning for the Construction of University Mathematics Microcourses

**DOI:** 10.1155/2022/6860842

**Published:** 2022-06-30

**Authors:** Yan Qiao, Haiming Fu

**Affiliations:** Guangzhou Huaxia Vocational College, Guangzhou, China

## Abstract

Outcome-Based Education (OBE) is a goal-based educational system in which each part of education is around outcomes. By the end of the course, every student should have achieved the goal. Outcome-Based Education (OBE) involves various teaching methods and is not restricted to any specified way of teaching. Based on the targeted results, the teacher will mentor the students by acting as an instructor, trainer, and facilitator. The Deep Learning Technology of Artificial Intelligence is applied in various applications to carry out automation and physical tasks without human intervention along with data transfer through wireless networking. In this research, an Apriori Algorithm supports the identification of a suitable method for the teaching process (the OBE Teaching concept) through the outcome of the learning process. This optimization of identification of suitable method is performed with the implementation of Ant Colony Optimization (ACO) in the construction of the University Mathematics Course. The study results proved that the proposed algorithm provides an accuracy of 98.87%. The proposed algorithm can be trained further based on different rules to attain some increased performance of the methodology.

## 1. Introduction

Outcome-Based Education (OBE) is a goal-oriented theory. Each student should have met their objective at the conclusion of their schooling. Rather than having a single method of instruction or evaluation, OBE classes, opportunities, and assessments should all work together to help students meet their goals. Faculty's function shifts from teacher to trainer to facilitator to mentor depending on the goals being sought [1]. As a reaction to the urgent need for educational reform, a number of initiatives have been launched. It was created in the 1950s to assist students to adapt to new challenges, adjust to technology developments, and utilize their knowledge in new settings for the benefit of society [2]. On the basis of a specific set of educational objectives, OBE is a typical approach to education. As students' progress through their education, they are tasked with meeting a variety of learning objectives and outcomes, both of which may be broken down into two categories: Programme objectives (PO) and Programme learning outcomes (PLO) [3]. While PLOs define what the students would be able to do after the completion of the program, POs identify the reasons or purpose of the programs. In practice, the POs of an OB academic program must meet the requirements of employers and other stakeholders and correspond with the institution's mission [4]. The PLOs specify the competencies the graduates must demonstrate based on POs. In this sense, a mapping relationship should be established between the program mission, POs, and PLOs. Students must also be taught and assessed in a way that enables them to achieve the stated goals of the PLOs in the curriculum, teaching and learning methodologies, and assessment strategies [5]. In engineering education, the professional bodies responsible for accrediting professional engineering, such as the Accreditation Board of Engineering and Technology, play a key role in hastening the shift towards the OBE paradigm. In Washington accord, an agreement of mutual recognition of programs between accreditation bodies of professional engineering has been taken place. However, academicians agree that despite the relevance of PO and PLOs for the design and certification of OB engineering programs, the words or their relationship to each other remain ambiguous [6]. Learning analysis (LA) has been more popular in tertiary education in recent years for a wide range of goals, including enhancing the learning process, improving feedback, enhancing learning experiences, and supporting decision-making. Association Rule Mining is a successful LA strategy (ARM). Discovering the connections between instructional information has been done using this method [7].

As a result, the goals or competencies students should display at the conclusion of their educational program define the curriculum material and organization, the teaching techniques and tactics, the course that is provided, the educational environment, or the evaluation methodologies [8]. Based on how to best attain the intended aim, all curricular and instructional options are developed. Implementing an outcome-based curriculum needs a sequence of steps: Learning objectives are clearly articulated in terms of content, context, and competency, and these goals are outlined in depth. The US Accreditation Council on Graduate Education has specified general competencies in patient care, medical knowledge, practice-based learning and improvement, system-based practices, interpersonal and communication skills, and professionalism [9]. Setting ‘benchmarks' for each step of the course is an excellent method to illustrate expected outcomes. The learner must be able to demonstrate the ability to complete each benchmark skill. Students should be able to demonstrate that they have met the curriculum's objectives at each level of study through the use of benchmarks. Content and teaching techniques are the third phase [10]. There are ‘Wholeclass models' that try to bring all students to high levels of learning before moving on, and then there are ‘Flexible models' that utilize flexible grouping, continuous progress, technology tools, and instructional management to achieve OBE [11]. There are no other aspects, such as what is taught, the amount of time it takes the 10 learners to obtain the outcomes, or whatever path they pick in order to realize their goals in OBE [12]. Students' portfolios and continuous assessments, both of which provide ongoing feedback between the student and the lecturer, would be extremely helpful in evaluating OBE [13]. Standard-referenced assessment may also be employed in OBE, which is a more precise type of criterion-referenced evaluation. The application of OBE is all students are capable of learning and can achieve high levels of competency when teachers delineate their expectations.

Numerous industries, including medical, business, robotics, and computer vision have already benefited greatly from data analytics. This growth in educational data has led to three new research fields: Educational Data Mining, Learning Analytics (LA), and Academic Analytics, which are all concerned with using computerized methods to analyze large collections of educational data that would otherwise be impossible or difficult to analyze [14]. While the three fields share the common goal of improving educational practice using data-driven approaches, several differences between them in their focus and the scale of analysis have been emphasized [15]. While LA focused on improving educational outcomes and applied to the data at the course, subject, program, and department levels, AA focused on improving educational results and applied the data at the institution, region, national, and international levels. EDM techniques, on the other hand, are applied to the data at any level because it focuses on the extraction of useful insights from of learning related data. Regardless of the difference between LA and EDM, the following are instances of important literature [16]. Program-related data of various types are evaluated using various data analytics approaches in each task to get insights into various elements of the program. If, for example, a survey of student learning outcomes is used to gather data, and experts' previous knowledge and neural network analysis are used to anticipate and assess student learning outcomes of an academic program and improve teaching quality [17]. Using a dataset from the catalogue of business programmes, a K-means clustering technique was used to analyze the association between business program competencies and the program title. Only a few programs have labels that do not accurately reflect what students will study [18]. At the learning object, module, and program levels, data analytics tools are utilized to find commonalities between course materials [19].

Traditional teaching and learning methods were contrasted to OBE structure and technology-aided education in terms of their impact on student academic progress in terms of GPA [20]. OBE students that used assistive technology had much higher average grade point averages than non-OBE students, according to the findings [21]. The average grade point average of OBE cohorts is much higher than that of non-OBE cohorts. For the purpose of ascertaining whether or not these schools have made the shift from instruction focused on processes to instruction focused on outcomes. The researcher used illuminative evaluation methods to examine the “matches” and “mismatches” between what was planned in an OBE text and what “actually happens” in classroom teaching [22]. Document analysis and naturalistic observations with follow-up probing interviews were used to gather data on how instructors intended to teach percentages and how they actually taught them in classrooms [23]. Educators' opinions were sought through a questionnaire before the findings were published. Five patterns were found: one that exclusively followed the OBE teaching plan, two that were more or less in accordance with the OBE text, and two that deviated from the OBE teaching plan. There were 58 percent of instructors who had changed to OBE and only 42 percent of educators who had not, according to the findings of the research [24]. Additionally, the survey revealed that educators choose to forego conceptual explanations in favor of “guided examples, group work, and reporting back,” teacher and student assessment, and ending tasks rather than teaching mathematics conceptually first. The study's primary recommendation was that instructors reclaim teaching mathematics conceptually before finishing examples and providing students with assignments [25]. Only a small percentage of the nation's math teachers have adopted the OBE method six years into the national innovation program. This study focused on OBE in the context of teaching math at the university.

## 2. Proposed Method

Mathematics is a vast subject with numerous areas like basic math, algebra, calculus, discrete mathematics, applied mathematics, computational mathematics, etc. Nowadays, top universities across the globe provide education online through distance education. They also offer various short-term courses in specified areas of mathematics, termed microcourses. These microcourses are educational courses conducted online and provide digital certification on course completion. In the current years of the Internet era, Mobile Learning and Online Education have reached almost every student. Top universities offer these microcourses with reasonable fees or free in some cases. The microcourses in Mathematics will be in a specific area of university mathematics, such as applied calculus, introduction to probability, algebraic studies, etc., to name a few. A course-providing website hosts these courses. This company will provide courses from all universities. With a paid subscription, students can access paid courses and free courses.

The course duration of these microcourses is concise compared to that of the full-time courses offered in regular courses. The microcourses will be in the form of videos and interactive apps. Students can select microcourses from their area of interest. In some cases, employed people look for microcourses in a specific area related to their work. In this way, the microcourses are customized to students and aspirants. Microcourses are accessed from anywhere and anytime with the Internet and are based on Artificial Intelligence like Deep Learning Technology. There is no time constraint in this type of education. The course itself can be self-paced, depending on the end users/students.

Moreover, the fee structure will be moderate. The limited version of the specified microcourse is free, and the unlimited version will come in the paid module. In some courses, the certificate of course completion also depends on limited/unlimited versions of the course provided. Some students prefer to study specified topics, similar to personalized courses. This fraternity will be benefited from the microcourses. The primary type of course material is a video tailor-made by the university. This video features critical points based on its importance to fit in the short duration of the course. Unlike a traditional classroom, this provides more concentration and saves a lot of time. If the students miss attending a class in conventional classrooms, they will miss the knowledge taught. In this case, students can access any number of repetitive times until he understands, with the help of artificial intelligence technology. With Deep Learning Technology, the AI identifies the student's understanding level, and replies are given based on their feedback comments. Students learn and understand the concepts deeply with the help of Deep Learning Technology.

Figure 1 represents the processes involved in the OBE teaching in higher education in promoting research in the mathematics course with the implementation of microcourses. This promotion of the course is achieved with the aid of wireless networking to make data transfer (video record of microcourses) from the teacher as one node to the students as multiple nodes. The data transfer occurs through the interactive system like mobile phones, laptops, and others that support uninterrupted Internet connection. Students, with their user credentials, can log in to the scheduled classes and undergo the course. After the course completion, the intelligent server will forward the feedback form to the students. Depending on the reply received, the quality of OBE is assessed and effective measure is taken.

Figure 2 represents the actual procedure involved in online teaching. The motive is to attract the students to the OBE Learning method in taking online courses. Online sessions are a part of the third-party accessing tool, and the universities imagine their students only to understand similar concepts given in their academic books. It might be a better idea to develop a separate team and create the online concepts. Without getting help from a site/web page or an application, it is challenging to reach children worldwide. The clarity of the concepts should be a focus in teaching. By organizing the teachers, the students can understand the subjects with systematic functionalities and many creative ideas to explain a concept. Students expect the teacher to relate the topic with any real-time applications, but it happens only very few times and only from a minimum teaching person.

### 2.1. Proposed Work

To motivate large scale innovation but also OBE, the Central Committee's Standard Presented in the following opinions just on the execution of Program Educational Objectives (PEOs) and Specific Outcomes (SOs) on developing innovation using the Ant Colony Optimization (ACO) Algorithm with Wireless Sensor Networks (WSN) but also Artificial Intelligence (AI). In this research, the WSN module plays a role in the data transfer from the server to the client and in collecting through the online evaluation system and the feedback form. This model has been used in higher education institutions to implement the Result Education or Outcome-Based Education (OBE) policy. Institutions of higher learning should incorporate students' OBE needs into society's imaginative needs, according to state organization's guidelines for innovation and OBE. Based on the school's attitude, this incorporation will define academic objectives. An Outcome-Based (OB) educational user's Program Outcomes (POs) should satisfy the specifications and bring out new teaching programs with OBE but also innovative thinking as themes. Equation (1) can also be deduced from the overall society knowledge but rather specific features of the time.

### 2.2. Apriori Algorithm Steps

Let *E*, the mission data, be a collection of data processing, with each transaction *x* consisting of a set of items denoted by *N* id. Let *s* = *s*_1_, *s*_2_,…, *s*_*m*_ represent a collection of things. A *v*-item set is one that contains *v* items. If a *v*-item set meets the minimal support requirement (Min sup), that is a frequent *v*-item set, indicated by *N*_*v*_. First, the Apriori Algorithm produced a collection of candidates, indicated by *N*_*v*_, which are candidate v-item sets. If the candidate item sets meet the minimum support requirements, they are frequent item sets. The algorithm is shown in Figure 3 and is discussed in detail below.

1. Assume a minimum confidence level (Min_sup) and just a minimum level of confidence (Min conf).
2. Scanning the dataset, potential *s*-item sets, *n*1, and determining the frequency of each item. The collection of infrequent *s*-item sets, *v*1, is next found, comprising the candidates' *s*-item sets in *n*1 with the lowest support. To produce candidate *s*-item sets, the technique employs *n*1.
3. Scanning the information again, infrequent 2-item sets, *v*2, are then identified, comprising candidate 2-item sets in *C*2 with the lowest supported. *v*2*v*2 then generates candidate 3-itemsets, *n*3.
4. Search the dataset again, check the minimum support of every contender in *ns* − 1 to Min sup, but then produce *ns* − 1, join *ns* − 1 *ns* − 1 to produce ns until it is no further eligible bulk productions are found.

To locate the frequent items, a two-step approach is used: combine then prune activities. (a) The joining procedure: If membership *s*1 but also *s*2 are joined, *ns* is formed by merging *ns* − 1 with itself to find *vs*.

The pruning procedure is as follows: Components of ns might not be common. A search of the database to ascertain the quantity of each possibility in *ns*, followed by the usage of *vs* − 1 to delete a contender *k*-item set in *ns*, will yield *vs*.

Its Apriori option start generating method decreases the size of item sets in so many circumstances. Nevertheless, if processing a large number of databases, the Apriori Algorithm may yield too many candidates for frequent item sets, so the programmer must scan the library frequently while looking for frequent item sets. This will take more resources and time to complete a single scan. As a result, it has to be efficient, as in the following equation:

(1) $$\begin{array}{c} {\text{Aprioris}}_{mu}=Ex_{s2x}^{\text{min}\_\text{sup}}N\left(n_{O};N:s,n^{*}\right)+s_{m}s=s_{1},s_{2},\ldots ,s_{m}\\ \text{ACO}s=Ex_{s2n}^{\text{min}\_\text{sup}}N\left(s:u_{O};N_{v};n^{*}\right). \end{array}$$

### 2.3. ACO Algorithm Steps

The organic behavior of ant colonies is inspired ACO algorithms. ACO has indeed been effectively applied to various difficult optimization issues, such as the Travelling Salesman Problem (TSP). Artificial ants were simple entities that use productive heuristics. The main principle behind constructively algorithms is to progressively construct solutions by contributing a resolution component to the partial solution in each phase until a whole product is implemented. Cooperation is a vital component of ACO algorithms since effective solutions are really the outcome of a collaborative interaction of multiple artificial ants throughout solution development. ACO has been used to solve a wide variety of difficult problem domains. Component but also phases, which seem to be combinations of constituents, are used to describe challenges. ACO Algorithm develops solution pathways in the field of these elements sequentially, adding additional elements to a condition. The ACO system is governed by two rules:

1. The rule of localized signal updating, which was used when building responses.
2. The global signal update rule, which has been implemented once all ants built a response.

Moreover, an ACO algorithm contains two trails suitable for usage: trail evaporating with, possibly, daemon operations. Trail evaporating reduces all path values immediately to protect the accumulation of tracks over a little component from becoming infinite. Disposable activities can also be used to accomplish centralized activities that single ants might do, such as invoking a local optimization technique or updating global information to determine whether it should bias its search strategy from such a nonlocal viewpoint.

Every ant evaluates a set of viable extensions to its present state at each step and advances to one in probability. The probability density function is described below. The likelihood of having to move from county *N* to system *u*_*O*_ for ant *N*_*v*_ is determined by the combination of discrete choices: the desirability of such move, as calculated by some optimization method denoting the Apriori attractiveness of such a move; and the trail level of a move, denoting how competent it has been in the past and make that specific move: it thus signifies a probability indication of the attractiveness of such a relocation, where

 
*u*_*O*_ and *N*_*v*_ are the sets of class
 
*v* is protected online class at a time, respectively,

where subscripts *N* are used to the number of infected and protected online classes until time *t*. At time ‘*v*,' just for notational simplicity, the source *s* can be estimated with the following equation implemented:

(2) $$\begin{array}{c} s_{m}=\sum_{n⟶0}^{s}Ex_{s2n}^{\text{min}\_\text{sup}}N\left(s\vdots u_{O};N_{t};n^{*}\right),\\ \text{ACO}s=\sum_{n⟶0}^{u}Ex_{s2n}^{\text{min}\_\text{sup}}\frac{N\left(u_{O};N_{v}\vdots s,n^{*}\right)N\left(s,n^{*}\right)}{N\left(u_{O};N_{v};n^{*}\right)},\\ {\text{Apriori}}_{s}=\sum_{s⟶0}^{n}Ex_{s2n}^{\text{min}\_\text{sup}}N\left(u_{O};N_{v}\vdots s,n^{*}\right).N\left(s¸\;n^{*}\right), \end{array}$$

where (Apriori_*s*_ and ACO*s*) seems to be from the Bayes' rule and *N*(*u*_*O*_; *N*_*v*_⋮*s*, *n*^*∗*^) has been the probability that the realizations *u*_*O*_ and *N*_*v*_ occur, provided an information source *s* and also the protector *n*^*∗*^. Thus, equivalent to if *N*(*s*, *n*^*∗*^) is uniformly distributed over equation (3), it detects whether or not a probability exists.

(3) $$\begin{array}{c} N\left(u_{O};N_{v}\vdots s,n^{*}\right).N\left(s,n^{*}\right)=\sum_{\sigma \in Ώ\left(s,n,u_{O};N_{v}\right)}N\left(\sigma |s,n^{*}\right). \end{array}$$

In which Ώ(*s*, *n*^*∗*^, *u*_*O*_, *N*_*v*_) denotes the full range of possible propagation sequences given *u*_*O*_; *N*_*v*_ and is represented in the following equation:

(4) $$\begin{array}{c} s_{mu}=Ex_{s\in u_{O}}^{\min\_\sup}N\left(s,n^{*},u_{O},N_{v}\right). \end{array}$$

The very same approach is used to determine the number of possible propagation sequences in the following equation:

(5) $$\begin{array}{c} s_{m}=Ex_{s\in u_{O}}^{\min\_\sup}N\left(s,n,u_{O},N_{v}\right).N\left(s,n^{*}\right), \end{array}$$

where

(6) $$\begin{array}{c} E\left(s,n^{*},u_{O},N_{t}\right)=\left|Ώ\left(s,n*,u_{O},N_{v}\right)\right|\\ =O\left(V+O\right)!\prod_{\mu \varepsilon I_{O}\cup^{}N_{v}}\left|V_{\mu }^{s}\right|-1. \end{array}$$

In equation (6), presumption for the set of possible propagation sequence nodes provides both information and context at the same time for *s*_*mu*_ and *s*_*m*_. It calls for *s*_*mu*_ and *s*_*m*_ in self-study reports distribution and consider |*V*_*μ*_^*s*^| be the number of programs where *n* and *s* are the information sources.

Put *I* in the center of the coordination system. *I* and *j* are two nodes that want to communicate about Entrepreneurship and Innovation (*Ex*).

Let *s* (*v*) be the network's set of nodes in the following equation:

(7) $$\begin{array}{c} \text{OBE}=\int s\left(v\right)=s\left(v-1\right)+\beta *m\left(v\right)\text{,}\;\text{where}-1\leq \beta \leq 1. \end{array}$$

*s*(*v*) represents the vertical and horizontal roads that might be fractious with each other at the connection. The mobile nodes are expected to move in front, *s*(*v* − 1) turn left or right, with a guaranteed connection. If *β* is less than zero, it means that the node is affected by deacceleration (negative acceleration) of residual battery energy (*E*) and consumed energy (*C*) of a node at time *t* as shown below:

(8) $$\begin{array}{c} \text{PO}s=\beta_{i\left(v\right)=}\sum_{i=1}^{v}\frac{E_{i\left(v\right)}}{C_{i\left(v\right)}}, \end{array}$$

(9) $$\begin{array}{c} NmO=\frac{\left(V^{i\;}mO\right)\beta }{\sum j\in O^{i}\text{PO}s\left(V^{i}jPOs\right)\beta },\beta \geq 1. \end{array}$$

If ∑*j* ∈ *O*^*i*^PO*s*(*V*^*i*^*jPOs*)*β* represents the current speed of the node is less than the minimum allowed velocity for its lane, then the current speed increases to *V*_min_ and is represented in equations (10) and (11). At long, last distinction of their speed is tolerable with OB being in respect to their positions and heading derived in equation (10).

(10) $$\begin{array}{c} \text{ifOB}=s\left(v\right)<s\text{maxThens}\left(v\right)=S\text{max,} \end{array}$$

(11) $$\begin{array}{c} \text{ifPO}s\left(v\right)<s\text{minThen}s\left(v\right)=S\text{min,} \end{array}$$

(12) $$\begin{array}{c} {\text{ACO}}_{s}=\sum_{j=1}^{i=1}V\left(i\right)\text{if}=s\left(v\right)<s\text{maxThens}\left(v\right)=S\text{max}. \end{array}$$

İn equation (12), ACOs is all about the number of student's responsibilities.

*s*(*v*) represents the student's language level objective; equation (13) represents distinction between the learner's cognitive stage and the level of difficulty with learning materials.

(13) $$\begin{array}{c} \text{OB}=Q_{i}\left(v\right)=\sum_{i=1}^{v}\frac{f_{i}O_{i}-s\left(v\right)}{g\left(v\right)-s\left(v\right)}. \end{array}$$

The smaller the difference *Q*_*i*_(*v*), the more closely the learning resource's expertise points match PO_*ij*_^*u*^(*v*) the learner's understanding points and are utilized as in the following equation:

(14) $$\begin{array}{c} {\text{Apriori}}_{s}=Ex_{i}^{u}\left(s\right)=\sum_{j\in u}PO_{ij}^{u}\left(v\right)+\text{OB}. \end{array}$$

The overall budget information between teaching materials is represented in equation (15) by PO*sEx*_*i*_^*u*^(*s*), the spending optimization problem with both educational resources.

(15) $$\begin{array}{c} \text{PO}s=Ex_{i}^{u}\left(s\right)={\left|v\right|}^{-0.6}\int_{-\infty }^{+\infty }V\left(\tau \right)p\left(\tau -x\right)e^{-jx\tau }V\tau . \end{array}$$

The primary purpose of the learning period *X*_*n*_(*u*) represents the objectives that highlight the differences in learning time required to complete the educational materials using *X*_*i*_*V*_*i*_(*s*)=*X*^*v*^*V*(*s*) and learning detection time as given in the following equation:

(16) $$\begin{array}{c} \text{SO}=L_{q}\left(s\right)=\sum_{i=1}^{Q}L_{i}E_{i}\left(s\right)=L^{E}E\left(s\right). \end{array}$$

The provisional license for the total optimization performance and OBE_*n*,*x*_ is the educational route created either by the comments thread function for calculating and comparing coefficients, as expressed by equation (17). It is a functional representation of the personalized learning route in the optimization technique.

(17) $$\begin{array}{c} {\text{OBE}}_{n,x}=\frac{N_{n,x}{}^{2}}{\delta^{2}}\int_{n=1}^{x=1}\left(\frac{\left(N_{n,x}*V\right)}{3\delta^{2}}\right)*\int \left[e^{i\left(N_{n,x}*V\right)}-e^{-\delta^{2}/3}\right]. \end{array}$$

The DL model is incorporated with the Apriori and the ACO to produce results with AI. The reason for incorporating both algorithms in this SL model is to identify whether the newly introduced teaching and learning methods are suitable for processes. In the case of AI, the intelligent system will automate the process of classifying the new teaching methods according to the outcome of the learning process.

## 3. Results and Discussion

The performance analysis of the self-study reports for the microcourses in the mathematics course is analyzed and the graphical representation of the same is given in Figure 3.

The study distribution taken for the duration of 2011 to 2020 is presented in Figure 4. In the initial years 2011 to 2013, it can be seen there is a good increase in the percentage of learning outcomes for the registered course. But later, from 2014 to 2020, the performance of the online self-paced course is in fluctuation. The numerical representation of this figure is given in Table 1.

From the definition of the Apriori Algorithm, if the candidate item sets meet the minimum support requirements, they are termed as frequent item sets. Later in the overall result analysis for the course, in Figure 5, a comparison of raw ACO and Apriori is considered. In Table 2, in any given university, the analysis of ACO and Apriori for certain subjects is considered. The analysis is performed based on the ACO number and the number of years the analysis is carried. The result percentage shows that the proposed model affects improved student learning through self-paced online resources. The percentage of learning accuracy increases with the incremental years. It can also be stated that with the support of updated technology, this progress in the results is achieved.

Equation (3) detects whether or not a probability exists; the analysis of the rule count is represented in Figure 6. The working principle of the Rule Count is the Rule-Based Algorithm of Machine Learning. The main role of this algorithm is to induce classification rules for the teaching and learning method classification in the training process. Frequency represents the number of counts a method obtained from the outcome of the learning process. It can be seen that as the frequency increases, the training & testing and accuracy performance have reached 95% approximately.  Table 3 represents the overall result obtained for the rule count based on the training and the testing frequency for ACO. Though the rule number changes with the antecedent and confidence count, the proposed algorithm provides better accuracy rate.

From equations (10) and (11), the current speed increases to *V*_min_ and is represented in analyses of ACOs and Apriori's in the statistical aspects which are represented in Figure 6. With the utilization of equation (16), the aspects considered for the statistical evaluation are the number of instances utilized, the number of programs conducted, the maximum, minimum, & average number of textual ACOs, and the most, least & average frequency of Apriori. From Figure 7 it can be observed that 680 numbers of instances are utilized, 150 numbers of programs or courses are considered for evaluation. The maximum, minimum, and average number of textual ACOs measured is as 150, 140, and 50, respectively. On the other hand, for the Apriori's frequency results, the most and least frequent results have reached approximately the same values. As the number of students and the programs is getting increased, the quantity analysis of ACO and Apriori will be increased gradually. The reason behind this increment is as the number of student nodes is updated in the network, the work of the intelligent system is also getting updated. All the results will be updated in the database or the server.

The performance analysis of the proposed Ant Colony Optimization algorithm with AI with the existing Apriori Algorithm is displayed in Table 4. Training and testing percentage refers to the percentage of successful training and testing processes. The ratio of the dataset used for training and testing processes is 80 and 20. However, accuracy is generally referred to as the validation accuracy of the model. The proposed algorithm has obtained an overall frequency of 185 which is higher than the Apriori Algorithm. The difference in the frequency analysis shows 58% increase in the proposed Ant Colony Optimized algorithm. Also, the training & testing and Accuracy results say that the proposed algorithm provides 5.22% and 2.53% increase over than Apriori Algorithm. The proposed algorithm can be trained further based on different rules and to attain some increased performance of the methodology.

## 4. Conclusion

OBE is an educational approach that is used to plan, evaluate, and acquire more knowledge for all students based on the achievement of unambiguous results and experiential learning. The implementation of the OBE approach in Mathematics subjects in universities is promoted in this paper, and students' motivation and learning are analyzed. Students' motivation and learning were assessed using an Ant Colony Optimization algorithm with WSN in this study. For teaching mathematics for learning and motivation, the algorithm works well. It is highly recommended that future studies examine the impact of university microcourses with OBE.

## Figures and Tables

**Figure 1:** Overall OBE teaching concept with microcourses.

**Figure 2:** Core Processes involved in learning.

**Figure 3:** Apriori Algorithm for OBE.

**Figure 4:** Performance analysis for the self-study reports distribution on over the years (2011–2020).

**Figure 5:** Analysis for the raw ACOs and Apriori dataset for the years (2011–2020).

**Figure 6:** Analysis of the Rule Count based training and testing Frequency in ACOs dataset.

**Figure 7:** Statistical aspects Frequency of ACOs and Apriori dataset.

**Table 1:** Result analysis for the self-study reports distribution over the years (2011–2020).

Years	Self-study reports distribution
2011	25
2012	30
2013	45
2014	35
2015	55
2016	45
2017	60
2018	79
2019	58
2020	60

**Table 2:** Overall Result Analysis for the raw ACOs and Apriori dataset (2011–2020).

	Programs	Years	ACO-No	Overall result per year in ACO text (%)	Overall result per year in Apriori_*s*_ (%)
University	1. Mechanical engineering	2011	1–3	85	86
		2012	1–4	80	82
		2013	1–3	82	83
	2. Civil	2014	1–3	84	82
		2015	1–4	92	87
	3. Management	2016	1–4	89	91
		2017	1–3	78	82
	4. Computer science	2018	1–3	83	88
		2019	1–4	93	91
		2020	1–3	95	94

**Table 3:** Overall Result for the Rule Count based training and testing Frequency in ACOs dataset.

Rule no	Count (antecedent)	Count (confidence)	Frequency	Training and testing (%)	Accuracy (%)
3456	184	0.62	134	78	92
3457	184	0.62	82	96	89
3458	184	0.62	62	75	92
3459	184	0.62	91	92	95
3460	184	0.62	81	89	93
3461	45	0.62	137	92	96
3462	45	0.62	78	95	90
3463	45	0.62	127	91	94
3464	45	0.62	212	96	96
3465	45	0.62	64	98	97

**Table 4:** Comparison of result frequency analysis of ACOs-Apriori for existing methods.

Algorithm	Overall frequency analysis of ACOs-Apriori	Training and testing (%)	Accuracy (%)
Ant Colony Optimization algorithm with AI	185	97.56	98.87
Existing method: Apriori Algorithm	127	92.34	96.34

## Data Availability

The data used to support the findings of this study are available from the corresponding author upon request.
